# Prognostic significance of DAPK promoter methylation in lymphoma: A meta-analysis

**DOI:** 10.1371/journal.pone.0210943

**Published:** 2019-01-25

**Authors:** Hong Wang, Lin-Yu Zhou, Ze-Bing Guan, Wen-Bin Zeng, Lan-Lan Zhou, Ya-Nan Liu, Xue-Yi Pan

**Affiliations:** 1 Department of Hematology, The First Affiliated Hospital of Guangdong Pharmaceutical University, Guangzhou, Guangdong, People’s Republic of China; 2 Department of Cardiology, The Third Affiliated Hospital of SUN YAT-SEN University, Guangzhou, Guangdong, People’s Republic of China; National Cancer Center, JAPAN

## Abstract

We aimed to characterize the clinical significance of epigenetic loss of death-associated protein kinase (DAPK) gene function through promoter methylation in the development and prognosis of lymphoma. PubMed, Web of Science and ProQuest databases were searched for relevant studies. Twelve studies involving 709 patients with lymphoma were identified. The prognostic value of DAPK methylation was expressed as risk ratio (RR) and its corresponding 95% confidence interval (CI), while the associations between DAPK methylation and the clinical characteristics of patients with lymphoma were expressed as odd ratios (ORs) and their corresponding 95% CIs. Meta-analysis showed that the 5-year survival rate was significantly lower in lymphoma patients with hypermethylated DAPK (RR = 0.85, 95% CI (0.73, 0.98), P = 0.025). Sensitivity analysis demonstrated consistent result. However, no associations were found between DAPK methylation and clinicopathological features of lymphoma, in relation to gender (OR = 1.07, 95% CI (0.72, 1.59), P = 0.751), age (OR = 1.01, 95% CI (0.66, 1.55), P = 0.974), international prognostic index (OR = 1.20, 95% CI (0.63, 2.27), P = 0.575), B symptoms (OR = 0.76, 95% CI (0.38, 1.51), P = 0.452), serum lactate dehydrogenase (OR = 1.13, 95% CI (0.62, 2.05), P = 0.683), and BCL-2 expression (OR = 1.55, 95% CI (0.91, 2.66), P = 0.106). Lymphoma patients with hypermethylated DAPK are at risk for poorer 5-year survival rate. DAPK methylation may serve as a negative prognostic biomarker among lymphoma patients, although it may not be associated with the progression of lymphoma.

## Introduction

Lymphoma accounts for about 3.6% of all cancer-related deaths in the developed countries [1]. It is a highly heterogeneous hematological malignancy that arises from the lymphatic system. Lymphoma patients exhibit wide range of responses to treatments and clinical outcomes [2–4]. At present, the international prognostic index (IPI) based on clinical parameters is widely applied to predict clinical outcomes. However, the variability observed in the patients’ outcome with similar clinical presentations undermines its prognostic value. However, the variability observed in the patients’ outcome with similar clinical presentations undermines the prognostic value of these factors in lymphoma [2–4]. Therefore, in order to improve the outcome prediction and indicate the requirement for aggressive therapy in patients with lymphoma, it is essential to identify effective prognostic biomarkers.

Recent studies showed that epigenetic modification, in association with aberrant methylation of deoxyribonucleic acid (DNA), can contribute to lymphomagenesis and cancer progression [5–8]. These aberrant methylations occur in the CpG (cytosine-phosphate-guanine) islands of the promoter region of tumor suppressor genes, repressing the level of gene transcription, leading to deregulation of cell pathways, including apoptosis, DNA repair, and cell cycle regulation, thus promoting tumorigenesis [7]. Death-associated protein kinase (DAPK) is a tumor suppressor, acting as a positive regulator of cell apoptosis. The loss of DAPK expression was first reported in cell lines derived from various human neoplasms including B cell neoplasms, bladder, breast, and renal cell carcinomas [9]. It was then discovered that the loss of expression was attributed to hypermethylation of the DAPK promoter region, resulting in gene silencing. Further analysis detected DAPK hypermethylation in 26% of tumor biopsy samples from colon cancer patients [10]. Subsequently, more studies reported the detection of DAPK promoter methylation in various human cancers [11]. For example, hypermethylation of the DAPK promoter was detected in 74 out of 107 cases with gastric cancers [12]. The methylated cases were correlated with a poorer, event-free survival [12]. Recent meta-analysis performed by Jia *et al*. showed that DAPK methylation levels were significantly higher in gastric cancer patients in the advanced stage and with lymph node metastasis, suggesting that DAPK methylation may be involved in the progression of gastric cancer [13]. In another study involving lung cancer, DAPK hypermethylation was detected in 59 out of 135 cases [14]. The methylated cases also showed poorer 5-year survival rates compared to those in unmethylated cases [14]. No correlation between DAPK methylation and tumor stage and histological subtypes were reported.

Epigenetic silencing of the DAPK gene through promoter methylation has also been observed in lymphoma [15]. Rossi *et al*. detected DAPK promoter methylation in 17 out of 20 patients with follicular lymphoma, 8 out of 11 patients with MALT lymphoma, and 71 out of 126 patients with DLBCL [15]. However, the clinical prognostic value of DAPK promoter methylation in lymphoma patients has been controversial. Several studies demonstrated that DAPK promoter methylation had no impact on the overall survival of lymphoma patients [16–21] while others associated DAPK hypermethylation with poorer overall survival [22–25]. In addition, the correlations between DAPK promoter methylation and clinicopathological parameters of lymphoma are also unknown.

Therefore, our present study aims to evaluate the effect of DAPK methylation on the 5-year mortality in patients with lymphoma and to investigate the clinicopathological significance of DAPK methylation in patients with lymphoma.

## Methods

This study was conducted in accordance with the PRISMA (Preferred Reporting Items for Systematic Reviews and Meta-Analyses) [26] guidelines. All analyses were based on previous published studies. No ethical approval or informed consent is required.

### Literature search strategy

A systematic search was conducted on PubMed, Web of Science, and ProQuest databases for relevant cohort studies published from inception to January 2017. The keywords used were (DAPK or DAPK1 or "Death-associated protein kinase" or "Death-associated protein kinase 1") AND (lymphoma or lymphoadenoma or adenolymphoma or "lymph-gland tumour") AND (methylation or methylated or demethylation or Hypermethylation or Hypermethylated).

### Literature screening

The identified articles were screened based on pre-set inclusion and exclusion criteria, sequentially starting from title, to abstract, followed by full text. Two researchers performed the screening concurrently, but independently. After completing the screening, the results were compared. When differences in the results were found, extensive discussion was then carried out between the researchers. When the differences could not be resolved through discussion, the opinion of a third researcher was sought in a group discussion until a consensus was reached.

### Inclusion criteria

Studies included in the meta-analysis all adhered to the following criteria:

1. Selected articles presented a comparison of DAPK methylation levels in patients with different clinical features of lymphoma.
2. Study subjects consisted of patients with lymphoma, not including lymphoid leukemia and other types of blood cancer.
3. The study outcomes included general clinical features as well as 5-year survival rates.
4. For duplicated studies, a single article was chosen based on comprehensiveness and the quality of reported outcome measurements.
5. All literature incorporated in the meta-analysis was published in English language.

### Exclusion criteria

The following studies were excluded:

1. Letters, excerpts, and reviews were excluded.
2. Articles that did not contain the required outcome measurements were excluded.

### Data extraction of articles

Two researchers independently extracted data from the aforementioned databases. The extracted data includes the author, year, country, diagnostic criteria, type of disease, number of patients, sample source, methylation detection method, clinicopathological parameters, patient 5-year survival rate, outcome, and follow-up. If the only available survival data were presented via Kaplan-Meier curves, we used Engauge Digitizer 4.1 to extract the mortality rates at 60 months (5-year). Each point was extracted 3 times in order to obtain an average value. Whenever discrepancies arose, the opinion of a third researcher was sought in a group discussion until a consensus was reached.

### Outcomes of interest

The primary outcome is 5 year mortality of the patients, which is derived from overall survival; secondary outcomes are the association between DAPK methylation and clinicopathological features of lymphoma, including gender, international prognostic index, B symptoms, serum lactate dehydrogenase, and BCL-2 expression.

### Quality assessment

The Newcastle-Ottawa Scale (NOS) was used to assess the methodological qualities of observational studies. The NOS consists of the following 3 categories: Selection (4 items), Comparability (1 item), and Outcome (3 items). A maximum of one star (*) is awarded to each item within the Selection and Exposure categories, and a maximum of two stars are awarded for Compatibility. The NOS score therefore ranges from 0 (worst) to 9 (best) stars. A high quality study was defined as one with a score of more than 5 stars.

The Quality in Prognosis Studies (QUIPS) tool was further used to assess the risk of bias in prognostic factor studies [27]. The QUIPS evaluates the risk of study bias in six domains: study participation, study attrition, prognostic factor measurement, outcome measurement, confounding measurement, and statistical analysis and reporting. Each domain was classified as low, moderate, or high risk of bias.

### Statistical analyses

All statistical analyses were performed using Stata 12.0. Dichotomous variables were analyzed by meta-analysis to study the association between DAPK methylation and the five-year survival rates or the varying clinical characteristics of lymphoma patients. Data on the predictive ability of DAPK methylation in patients with lymphoma were pooled using risk ratio (RR) and its corresponding 95% confidence interval (CI) for 5-year mortality, while the associations between DAPK methylation and various types of clinical characteristic of lymphoma patients were expressed in the form of odds ratios (ORs) and their 95% CIs.

Heterogeneity was assessed statistically by the Cochran’s Q test and I^2^ test (I^2^ = 0–25%, low heterogeneity; I^2^ = 25–50%, moderate heterogeneity; I^2^ = 50–75%, large heterogeneity; and I^2^ = 75–100%, extreme heterogeneity). When significant heterogeneity between studies was identified (P value for Cochran’s Q test <0.1 or I^2^> 50%), the random-effects model was applied. In other cases, the fixed-effects model was used to calculate the pooled estimates accordingly.

To further assess the influence of selected studies on the pooled results, leave-one-out sensitivity analysis was performed by omitting each study in turn to confirm that findings of the current meta-analysis were not driven by any single study. If the point estimate of its omitted analysis lay outside the 95% CI of the combined analysis, it was indicative that the removed study had an impact on the overall estimates and that the pooled results are not robust. No assessment of publication bias was done in the present study as tests for funnel plot asymmetry are performed when at least 10 studies are included in a meta-analysis.

## Results

### Selection of studies

The initial screening of the literature yielded 220 research articles (PubMed 51, Web of science 43, ProQuest 126). 36 were duplicated studies and were removed using Endnote or manual deletion. The remaining 184 articles were preliminary screened by titles and abstracts. 158 articles were eliminated because they did not meet the screening criteria. 26 research articles underwent full text screening. 14 articles were further eliminated as they did not meet the eligibility criteria or consisted of repeated data. In total, 12 articles that studied the clinicopathological or prognostic value of DAPK methylation in patients with lymphoma were eventually included in the subsequent meta-analysis. The process utilized for filtering the literature is depicted in greater detail in Fig 1.

**Fig 1:** Flow diagram of study selection.

### Study characteristics and quality assessment

Twelve studies [5, 16–18, 20–24, 28–30] with a total of 709 patients were included for meta-analysis. Detailed characteristics of the included studies are depicted in Table 1. The included studies were published between 2006 and 2016. The studies originated from Asia (5), Europe (4), North Africa (2), and North America (1). Subjects included patients with DLBCL, cutaneous marginal zone B-cell lymphoma, follicular lymphoma, Hodgkin lymphoma, thymic and gastric MALT lymphomas, and primary central nervous system (CNS) and gastric lymphomas. Disease diagnoses were made based on World Health Organization (WHO) classifications. DAPK methylation was quantitated using allelic methylation-specific polymerase (MSP) chain reaction pyrosequencing or MSP assays on tissue or bone marrow samples.

**Table 1:** Characteristics of the included studies for prognostic or clinicopathological analyses.

Author, year	Country	Diagnostic criteria	Disease	Treatment	No.	Sample source	IPI (Low/High)	Age	Methylation detection method	Outcome	Follow-up
Munch-Petersen HD (2016)[16]	Denmark	WHO classification	DLBCL	Chemo- and immunotherapy, whole brain radiotherapy (WBRT) including number of fractions and dose ^1^	107	Tissue	27/55	64.2±1.2	Allelic MSP pyrosequencing	There was no significant difference between OS/PFS of patients with or without methylation of DAPK in the entire cohort.	9.2 months [95% CI: 4.0–14.4]
Takino H (2008)[17]	Japan	WHO—EORTC classification	Cutaneous marginal zone B-cell lymphoma	Treatments including surgical excision, topical steroid, psoralen and ultraviolet A phototherapy, and chemotherapy	60	Tissue	-	57(26–87)	MSP assay	Prognostic analysis showed that DAPK hypermethylation had no impact on the disease-free survival of the patients (data not shown).	36 months (7–18)
Takino H (2013)[21]	Japan	WHO classification	Thymic MALT lymphoma	Surgically resected with or without additional treatment (chemotherapy or radiotherapy)	18	Tissue	-	55(23–68)	MSP assay	Prognostic analysis showed that DAPK hypermethylation had no impact on the overall survival of the patients.	61.1 months (6–252)
Kristensen LS (2014)[24]	Denmark	WHO classification	DLBCL	R-CHOP-like regimens immunotherapy with rituximab	119	Tissue	80/39	59.8(22–90)	Allelic MSP pyrosequencing	Prognostic analysis revealed that the hypermethylation of DAPK genes was associated with a significantly poorer OS and DFS.	-*
Chu LC (2006)[28]	America	WHO classification	Primary CNS lymphomas	-	25	Tissue	-	64	Allelic MSP pyrosequencing	-	-
Manuela Giachelia (2014)[23]	Italy	WHO classification	Follicular lymphoma	Standard immunochemotherapy ^2^	107	Bone marrow	66/41	57(28–83)	Allelic MSP pyrosequencing	Prognostic analysis revealed that the hypermethylation of DAPK genes was associated with a significantly poorer PFS.	43 months (4–139)
Krajnovic M (2014)[18]	Serbia	WHO classification	DLBCL	Treated with rituximab in addition to the standard chemotherapy	51	Tissue	29/50	52.4(19–83)	Allelic MSP pyrosequencing	Prognostic analysis showed no significant difference in the OS between patients with hypermethylated and unmethylated DAPK.	30.5 months (1–111)
Dhiab MB (2015) [29]	Tunisia	WHO classification	Hodgkin lymphomas	-	53	Tissue	-	6–71	Allelic MSP pyrosequencing	-	-
Kondo T(2009) [30]	Japan	WHO classification	Gastric MALT lymphoma	-	21	Tissue	-	-	Allelic MSP pyrosequencing	-	-
Nakamichi I (2007) [20]	Japan	WHO classification	DLBCL	Chemotherapy ^3^	53	Tissue	40/13	65(23–91)	MSP assay	Prognostic analysis showed that DAPK hypermethylation had no impact on the 5-years survival rate of the patients.	24.6 months (7–146)
Amara K (2008) [22]	Tunisia	WHO classification	DLBCL	Chemotherapy ^4^	46	Tissue	33/13	65(18–85)	MSP assay	Prognostic analysis revealed that the hypermethylation of DAPK genes was associated with a significantly poorer OS and DFS.	15 months (0–96)
Huang Q (2007) [5]	China	WHO classification	Primary gastric	-	49	Tissue	-	51(15–77)	MSP assay	-	-

-*: Kaplan-Meier curves were provided, but values were not provided in study.

-: No follow-up information was provided.

^1^ Combination chemotherapy includes CNSBONN (patients<65 years: high dose-methotrexate (HDMTX), cytarabine, thiotepa, +/- rituximab, and ASCT (autologous stem cell transplantation), patients>65 years: methotrexate, vincristine, procarbacine +/- rituximab), carmustine+HDMTX, CNS IELSG (CHOP/CHOP-like regimens +/-HDMTX, cytarabine or alkylating agents+methotrexate), NORDIC CNS (CHOP-like regimen: rituximab, HDMTX, highdose-cytarabine, cyclophosphamide, iphosphamide, vincristine, vindesine, followed by temozolomide, and intraspinal depocyte), MVBPCNS (HDMTX, vincristine, carmustine, prednisolone), vincristine+HDMTX, all +/-rituximab. One HDMTX-treated patient was also treated with rituximab (survived 1251 days). In total, 70+1 patients 21/71 (29.6%) had rituximab. Of the whole cohort, 21/108 (19.4%) were treated with rituximab.

^2^ R-chemo, rituximab-based immunochemotherapy (rituximab, cyclophosphamide, doxorubicin, vincristine, and prednisone; rituximab, vincristine, and prednisone; and rituximab, fludarabine, and mitoxantrone).

^3^ Chemotherapeutic agents administered were cyclophosphamide, DXR or its analogues, vincristine andpredonisolone (CHOP or THP-COP) in 24 patients, CHOP or THP-COP and rituximab in 16, CHOP and VP-16 in four, CHOP, VP-16, and bleomycin in four, VP-16 alone in one, and other combination in four.

^4^ Ten (22%) patients have been treated with CHOP, eight (17%) with COP, 10 (22%) with ACVBP, seven (15%) with CVP, and 11 (24%) with mini-CEOP.

**Abbreviations**: DLBCL: diffuse large B-cell lymphoma; DAPK: death-associated protein kinase; MSP: methylation-specific polymerase chain reaction; MALT: Mucosa-associated lymphoid tissue; WHO: World Health Organization; OS: overall survival; DFS: disease-free survival; PFS: progression-free survival

The methodological quality of each of the 12 observational study was evaluated using the NOS. Seven studies [16–18, 20–23] had a score of 9 stars. The other five studies [5, 24, 28–30] lacked information in their outcome measurements and therefore had a score of 7 stars. Overall, these 12 studies were considered high quality studies (Table 2).

**Table 2:** Quality assessment of the observational studies based on the Newcastle-Ottawa Scale.

	Selection				Comparability	Exposure			Score
	Representativeness of the exposed cohort	Selection of the non exposed cohort	Ascertainment of exposure	Demonstration that outcome of interest was not present at start of study	Comparability of cohorts on the basis of the design or analysis	Assessment of outcome	Was follow-up long enough for outcomes to occur	Adequacy of follow up of cohorts	
Munch-Petersen HD (2016)[16]	*	*	*	*	*	*	*	*	9
Takino H (2008)[17]	*	*	*	*	*	*	*	*	9
Takino H (2013)[21]	*	*	*	*	*	*	*	*	9
Kristensen LS (2014)[24]	*	*	*	*	*	*			7
Chu LC (2006)[28]	*	*	*	*	*	*			7
Giachelia M (2014) [23]	*	*	*	*	*	*	*	*	9
Krajnovic M (2014)[18]	*	*	*	*	*	*	*	*	9
Dhiab MB (2015) [29]	*	*	*	*	*	*			7
Kondo T (2009) [30]	*	*	*	*	*	*			7
Nakamichi I (2007) [20]	*	*	*	*	*	*	*	*	9
Amara K (2008) [22]	*	*	*	*	*	*	*	*	9
Huang Q (2007) [5]	*	*	*	*	*	*			7

Among the 12 included observational studies, 6 studies [18, 20–24] also reported the prognostic value of DAPK methylation in patients with lymphoma. There were two studies, which are Munch-Peterson (2016) and Takino (2008), only reported the outcome or conclusion of prognostic value of DAPK methylation in patients with lymphoma, without providing sufficient information or data for analysis for prognostic value of DAPK methylation in patients with lymphoma. We assessed the risk of bias in these 6 prognosis studies using the QUIPS tool (Table 3). Five studies [18, 20, 22–24] were of low risk in all domains, while one study [21] was inadequate in its prognostic factor measurement and did not account for potential confounders in its study, resulting in the high risk of bias in 2 domains. All papers were generally good at reporting study participation, study attrition, outcome measurement, and statistical analysis and reporting, indicating a relatively high methodological quality in general.

**Table 3:** Quality assessment of the included studies based on the quality in Prognosis Studies tool.

	Study participation	Study attrition	Prognostic factor measurement	Outcome measurement	Confounding measurement and account	Analysis
	The study sample represents the population of interest on key characteristics, sufficient to limit potential bias to the results.	Loss to follow-up (from sample to study population) is not associated with key characteristics (i.e., the study data adequately represent the sample), sufficient to limit potential bias.	The prognostic factor of interest is adequately measured in study participants to sufficiently limit potential bias.	The outcome of interest is adequately measured in study participants to sufficiently limit potential bias.	Important potential confounders are appropriately accounted for, limiting potential bias with respect to prognostic factor of interest.	The statistical analysis is appropriate for the design of the study, limiting potential for presentation of invalid results.
Takino H (2013)[21]	Low	Low	High	Low	High	Low
Kristensen LS (2014)[24]	Low	Low	Low	Low	Low	Low
Giachelia M (2014)[23]	Low	Low	Low	Low	Low	Low
Krajnovic M (2014) [18]	Low	Low	Low	Low	Low	Low
Nakamichi I (2007)[20]	Low	Low	Low	Low	Low	Low
Amara K (2008) [22]	Low	Low	Low	Low	Low	Low

### Association between DAPK methylation and prognosis of lymphoma patients

Among the 12 studies included, 6 studies [18, 20–24] with a total of 362 patients analyzed the association between DAPK methylation and patients’ 5-year survival rates, mainly in patients with thymic MALT lymphoma [21], follicular lymphoma [23], and DLBCL [18, 20, 22, 24]. The results showed moderate heterogeneity between the studies (I^2^ = 45.7%, P = 0.101). The fixed-effects model showed that the 5-year survival rate was significantly lower in lymphoma patients with DAPK methylation than in patients without methylation (RR = 0.85, 95% CI (0.73, 0.98), P = 0.025) (Fig 2A). Sensitivity analysis showed that no individual studies significantly affected the pooled RR, indicating the stability of the result (Fig 2B). The statistically significant lower 5-year survival rate suggests that DAPK methylation might be a general, poor prognostic factor for lymphoma.

**Fig 2:** Association of DAPK methylation with 5-year survival rate in patients with lymphoma. (A) Forest plot (B) Sensitivity analysis.

### Association between DAPK methylation and the clinicopathological parameters of lymphoma patients

The correlations between DAPK methylation and the clinical features of lymphoma were summarized in Table 4. There were no significant differences in the DAPK methylation levels between the male and female patients (OR = 1.07, 95% CI (0.72, 1.59), P = 0.751) (Fig 3A) or between the young and old patients (OR = 1.01, 95% CI (0.66, 1.55), P = 0.974) (Fig 3B). The international prognostic index (IPI) score based on clinical parameters during presentation categorizes patients into low/low-intermediate or high/high-intermediate risk groups. Patients with lower IPI scores had no significant difference in DAPK methylation levels from those with higher IPI scores (OR = 1.20, 95% CI (0.63, 2.27), P = 0.575) (Fig 3C). There was no significant difference in DAPK methylation level among lymphoma patients with or without B symptoms (OR = 0.76, 95% CI (0.38, 1.51), P = 0.452) (Fig 3D). The methylation of DAPK in lymphoma patients with normal or elevated serum lactate dehydrogenase (LDH) and with or without BCL-2 expressions was also analyzed. The results showed that the degree of DAPK methylation in lymphoma patients with normal LDH levels was not significantly different from that of lymphoma patients with elevated LDH levels (OR = 1.13, 95% CI (0.62, 2.05), P = 0.683) (Fig 3E). DAPK methylation levels were also not significantly different between lymphoma patients with normal and abnormal BCL-2 levels (OR = 1.55, 95% CI (0.91, 2.66), P = 0.106) (Fig 3F).

**Table 4:** Overall analysis of the association between DAPK methylation and clinical features of patients with lymphoma or DLBCL.

Variables	No. of study	No. of lymphoma patients	RR/OR (95% CI)	P value	Heterogeneity	
					I^2^	P value
**Lymphoma**						
5-year survival rates	6	362	0.85 (0.73, 0.98)	0.025	45.7%	0.101
Gender	10	539	1.07 (0.72, 1.59)	0.751	33.6%	0.139
Age	9	535	1.01 (0.66, 1.55)	0.974	9.1%	0.360
IPI-score	4	283	1.20 (0.63, 2.27)	0.575	0.0%	0.502
B symptoms	3	214	0.76 (0.38, 1.51)	0.452	0.0%	0.794
LDH	4	260	1.13 (0.62, 2.05)	0.683	0.0%	0.486
BCL-2	4	272	1.55 (0.91, 2.66)	0.106	19.3%	0.293
**DLBCL**						
5-year survival rates	4	265	0.90 (0.62, 1.29)	0.557	70.3%	0.018
Gender	4	291	0.88 (0.48, 1.60)	0.675	0.0%	0.608
Age	4	288	1.09 (0.60, 1.99)	0.775	0.5%	0.389
IPI-score	4	283	1.20 (0.63, 2.27)	0.575	0.0%	0.502
B symptoms	3	214	0.76 (0.38, 1.51)	0.425	0.0%	0.794
LDH	3	214	0.95 (0.48, 1.89)	0.878	0.0%	0.488
BCL-2	2	102	3.49 (0.16, 74.37)	0.423	71.6%	0.060

**Fig 3:** Association of DAPK methylation with clinical features of lymphoma. (A) Gender (B) Age (C) International prognostic factor (IPI) (D) B symptoms (E) Serum lactate dehydrogenase (LDH) (F) BCL-2 expressions.

### Analyses of DAPK methylation in DLBCL patients

We further performed analyses to evaluate the role of DAPK promoter methylation in DLBCL patients. Analysis of 4 studies [18, 20, 22, 24] with a total of 265 patients showed that the 5-year survival rate in DLBCL patients with DAPK methylation was not significantly different from those without methylation (RR = 0.90, 95% CI (0.62, 1.29), P = 0.557) (Fig 4A). Sensitivity analyses demonstrated consistent results (Fig 4B). Our results indicate that that DAPK methylation is not associated with the progression of DLBCL. However, the result should be interpreted cautiously as there was statistically significant large heterogeneity between studies (I^2^ = 70.3%, P = 0.018).

**Fig 4:** Association of DAPK methylation with 5-year survival rate in DLBCL patients. (A) Forest plot (B) Sensitivity analysis.

Our results similarly showed no association between DAPK methylation and clinicopathological features of DLBCL, in relation to gender (OR = 0.88, 95% CI (0.48 1.60), P = 0.675) (Fig 5A), age (OR = 1.09, 95% CI (0.60, 1.99), P = 0.775) (Fig 5B), IPI (OR = 1.20, 95% CI (0.63, 2.27), P = 0.575) (Fig 5C), B symptoms (OR = 0.76, 95% CI (0.38, 1.51), P = 0.425) (Fig 5D), LDH (OR = 0.95, 95% CI (0.48, 1.89), P = 0.878) (Fig 5E), and BCL-2 expression (OR = 3.49, 95% CI (0.16, 74.37), P = 0.423) (Fig 5F). Results were summarized in Table 4.

**Fig 5:** Association of DAPK methylation with clinical features of DLBCL. (A) Gender (B) Age (C) International prognostic factor (IPI) (D) B symptoms (E) Serum lactate dehydrogenase (LDH) (F) BCL-2 expressions.

## Discussion

Six studies [18, 20–24] analyzed the association of DAPK methylation with 5-year mortality in patients with lymphoma. Our result shows that lymphoma patients with DAPK promoter methylation have poorer 5-year survival rates compared to those without methylation. Moderate but statistically insignificant heterogeneity was observed despite including studies involving various types of lymphoma, including DLBCL [18, 20, 22, 24], MALT lymphoma [21], and follicular lymphoma [23]. Sensitivity analyses showed consistent results, indicating that no individual study significantly affected the pooled result. Our result, therefore, suggested that DAPK hypermethylation could be a general pathological event in lymphoma and that it might be used as a prognostic biomarker among lymphoma patients.

We also analyzed the association of DAPK methylation with 5-year mortality in patients with DLBCL. Contrary to our 5-year survival rate analysis in all lymphoma patients, the 5-year survival rate in DLBCL patients with DAPK methylation was not statistically significant lower than those without DAPK methylation. However, this result has to be interpreted with caution because statistically significant large heterogeneity was present between studies. The limited number of studies and patients unable us to exactly identify the source of heterogeneity. Therefore, more studies are required to determine whether DAPK methylation can be used as a biomarker to predict poorer 5-year survival in DLBCL patients.

The DAPK gene, located on human chromosome 9q21.33, encodes a calcium/calmodulin-regulated serine-threonine kinase. It participates in the apoptosis-inducing pathways triggered by interferon γ, tumor necrosis factor-α, and the FAS ligand. Upon stimulation, DAPK activates p53 through direct phosphorylation and inhibition of mouse double minute 2 homolog (MDM2), a p53 inhibitor, promoting apoptotic signals. Recent studies have also suggested the involvement of DAPK in non-apoptotic cell death through autophagy, or through the formation of membrane blebbing [11, 31]. Therefore, the attenuation of DAPK functions through methylation could be one of the key mechanisms for cancer cells to evade cell death and promote chemo-resistance [32].

We also analyzed the correlations between DAPK promoter methylation and the clinicopathological features of lymphoma. Our findings show that DAPK promoter methylation is not correlated with gender. However, in a study by Kondo *et al*., the level of DAPK methylation in male patients was found to be significantly higher than that in female patients with gastric MALT lymphoma [30]. The susceptibility of male patients to DAPK promoter methylation specifically in gastric MALT lymphoma, therefore, requires further investigation. Analyses based on age did not show significant correlation, indicating that methylation of the DAPK gene is not influenced by an age factor. The age group in different studies has been inconsistent with division at 65 [5, 16, 24, 28, 30], 60 [17, 18, 22, 25], and 54 [29] years old. However, heterogeneity was not significant. Hence, it can be concluded that age division has an insignificant effect on the result. Interestingly, our data also revealed that methylation of DAPK is independently associated with the IPI score, B symptoms, serum LDH, and BCL-2 expressions. These clinicopathological parameters are often associated with the progression of lymphoma. Therefore, our results could implicate that DAPK methylation is not associated with the progression of lymphoma. Similarly, analysis of DLBCL studies indicated that DAPK methylation was not correlated with gender and age status. There were also no significant differences in the DAPK methylation levels between DLBCL patients with high or low IPI scores, B symptoms, or between the varying levels of serum LDH and BCL-2.

There are a few limitations in this study. Some of the included studies used the traditional MSP chain reaction method in the detection of DAPK methylation. MSP is an error-prone assay. The non-specific amplification of unmethylated sequences and the incomplete bisulfite conversion may generate false-positive results [19]. Therefore, the data collected through MSP might be less accurate. Additional pyrosequencing has been suggested to confirm all positive results. Moreover, the definitions of hypermethylation are different among studies. For instances, in the studies by Kristensen *et al*. [19, 24, 25], the hypermethylation is defined as the methylation levels being above two standard deviations from the control mean methylation level, while in the study by Giachelia *et al*.[23], the methylation levels that are higher than the upper limit of healthy controls are defined as hypermethylation. The variance in cutoff values may also introduce bias in our analysis. Additionally, extrapolation of the 5-year mortality rate indirectly from the Kaplan-Meier curve may be less accurate compared to acquiring directly from the original statistics. All of these factors could influence the interpretation of our results. Therefore, further studies with larger sample sizes involving all types of lymphoma, precise detection methods, and standardized definition of hypermethylation are warranted. Another limitation of the study is the use of unadjusted risk ratio and/or rates in estimating the effect of various variables on survival, which may introduce biases to the study.

## Conclusion

Lymphoma patients with hypermethylated DAPK are at higher risk of death within 5 years. However, our results did not support the association of DAPK methylation with increased 5-year mortality rate in DLBCL patients. Our analyses were limited by the number of studies, variability in methylation detection methods and our results were pooled using unadjusted data. Future high quality studies are warranted. Our results also showed that DAPK methylation is not associated with gender, age, IPI score, B symptoms, serum LDH, or BCL-2 expression. Our findings indicate that methylation of DAPK in lymphoma may serve as a prognostic biomarker in lymphoma, but not as an indicator for disease progression.

## Supporting information

S1 Checklist PRISMA checklist. (DOC)
